# Empirical Investigation on the Characteristics and Perceived Value of Patients in Medical Treatment Seeking: In-Depth Research in Zhejiang Province of China

This article has been retracted.

**DOI:** 10.1155/2021/5245041

**Published:** 2021-12-24

**Authors:** Hui Qian, Wu Lu, Daliang Zhang

**Affiliations:** ^1^Zhejiang University City College, Hangzhou 310000, China; ^2^Zhejiang University, Hangzhou 310000, China

## Abstract

**Background:**

Patient Perceived Value (PPV) provides a valuable perspective to explain why the government reforms on health system in terms of functional medical treatment performance improvement did not decrease the crowded waiting line or increased patient satisfaction in China.

**Methods:**

Questionnaires comprising seven constructs were sent to patients from seven highly recognized hospitals in Zhejiang Province of China. It was collected via face-by-face in a twelve-month period (2019), and 2586 valid data were collected for SPSS statistic accordingly.

**Results:**

Besides the significance of the functional medical treatment values (such as the treatment effectiveness, accurate price, standardization, and normalization), the emotional values (reasonable waiting time, convenient accessibility, communication with doctors/nurses) were significant in patients' consciousness. Patient medical treatment seeking preferences were affected by patients' background characteristics and perceived value, which consequently produced differentiated patients' satisfaction. Patients' characteristics, which related to the age, gender, illness conditions, educational, and income level, would have different demanding in medical treatment seeking. These young female patients in outpatient or in mild illness conditions with higher educational and income levels tend to be relatively high in timing and convenience demanding.

**Conclusion:**

This result would change the policy maker and hospitals to considerate the patients' emotional value as well as functional value in providing medical treatment. Classified patients' time arrangement tactics consistent with distinguished characteristics, equipped up with convenient accessibility and interconnected medical treatment environment design, can create valuable patients' satisfaction in China.

## 1. Background

After a two-decade national wide medical quality-inspired reconstruction and health care reform in China, the quantity and violence level of medical conflicts still remained as a representative form of social contradictions [1, 2]. Medical treatment is characterized by unpredictable risks and difficulty, which could be a costly burden for patients under current inequitable and inefficient social insurance program in China [2, 3]. However, the unbalanced medical expertise and resource allocation drive patients flow to wide recognized hospitals in big cities and thus make medical treatment seeking experiences worse [3, 4].

Patient satisfaction generally reflected the quality and performance in hospitals as an essential improvement indicator [5]. There are varied reasons identified by researchers for patients' dissatisfaction, and the functional value of medical treatment was believed as the key value which originated from the normalization and quality [6]. Research studies based on structure-process-outcome analysis expanded the assessment of the medical service quality from patients' perspectives: “structure” indicated the environment and physical facility in hospitals, “process” implied the treatment experiences in interacting with hospital staffs, and “outcomes” meant the physical treatment consequence and psychological impression during the interactions [7]. Medical incidents and disputes destroyed public trust and impaired hospitals' reputation. It implied nontransparent treatment details, or unclear treatment processes could result in untrustworthiness, which would largely enlarge the medical disputes and patient-doctors' conflicts in China.

Researches also displayed, especially in big public hospitals, patient dissatisfaction was mainly occurred on the doctor-patients' and nurse-patients' communication and interaction, rather than medical treatment technique quality only [8, 9]. A report pointed out that 82% patients' dissatisfaction were mostly due to limited information they received, 67% were the result of doctors' and nurses' indifference in communication, 63% were unhappy with medical treatment accurateness, and 44% were the little chance to ask problems without restraint [10]. Additional study also showed a similarity result that 73% of patients did not trust their doctors with only 8% who specified that they completely trust their doctors because of inadequate communication [11].

Accessibility and effectiveness, besides of the quality of the medical treatment techniques, were highly valued by patients and reflected the service capacities of doctors as well [5, 12]. An investigation in a famous hospital in Beijing found that the workload of doctors exceeds 200 patients per day, which leaves one patient waiting for hours for treatment [13]. Waiting time and medical treatment convenience were the additionally significant sources of dissatisfaction, asides from treatment quality [14]. Any unintended postpone and unpleasant interaction will intensify patients' untrustworthiness and dissatisfaction.

Nonetheless, few quantitative studies in Chinese hospitals systematically investigated patients' characteristics and their differentiated perspective values. These results led to growing researches on managing satisfaction and relationship levels to patient' perspective value analysis. Further in-depth research would be worthful to expand the hospital management and health care reform system study in China.

## 2. Literature Review

Medical disputes happened due to the gaps or differences between hospitals and patients' expectations about the medical treatment satisfaction [7]. Traditionally, one of the main factors influencing satisfaction rate concerned the medical expenses [15]. While low medical expenses reduce the patient's financial burden, a high medical fee might lead them to believe they are overcharged for unnecessary examination and the types of drugs prescribed. Patients would struggle with worried, anxious, and tired while waiting for medical treatment. These stressing moods eventually shape their medical seeking experiences and even treatment effectiveness [16]. A qualitative study revealed that functional value, emotional value, and social value in patients' value system could be, respectively, analyzed in satisfaction assessments [17]. However, the satisfaction in patients' value remained unpredictable, and doctor-patient relationships could be associated with varied factors [9].

PPV gave a critical argument that if patient satisfaction is the result from doctors' medical skill and service quality [14, 18]. It armed to clarify why developed medical techniques and capability still leaved a high rate of dissatisfaction and a low level of patients' loyalty and satisfaction [18, 19]. Patient Perceived Value (PPV) is reflected by an integrated assessment about the received values against expectations on the medical service utility from patients, which is the development of the theory of customer perceived value in the medical field [20].

Several dimensions were extended into more detailed constructs, covering technique professionalism and normalization, service and facility quality, accessibility, convenience, social reputation, patient-doctor relationships, treatment cost and control, etc. [21, 22]. The government of China launched series of regulatory changes to enhance doctors and nurses' work normalization.

When considering patient-doctor relationship as one crucial foundation of patient retention, PPV highlighted the quality of medical information sharing and patient-doctor communication [20, 23–26]. Patients gave a high value to an adequate communication which emphasized a shared decision-making model between doctors and patients [10]. Based on patient's understanding language, knowledge, values, and preferences, these predictable benefits and drawbacks of treatment alternatives should be clarified [14, 18]. But the reality in Chinese hospitals was the overloaded work time and unequaled motivation system caused doctors dissatisfied and negative emotions convey to patients [15]. Afterwards, prejudice and impression of unprofessional and unqualified destroyed patients' trust of doctors and their treatment decisions.

Additionally, another keystone in guiding patients' decision in medical treatment seeking is the public reputation. Patients' tension about high self-paying drugs or medical treatment expenses would be positively released by the high esteem of hospitals or famous doctors, but otherwise, would be expected as overtreatment and overprescription [6].

Convenience, comfortable environment, and faster assess related to the treatment surrounding could foster more relaxed emotion, accompanied by fairness and efficiency perceptions [6, 16]. Delays in the appointment due to the number of patients increased the tensions and conflicts [1]. The dissatisfaction led many Chinese hospitals to adopt IT systems to improve patient convenience and workflow efficiency. These e-programs in hospitals, such as electronic registering machine, electronic health record (EHR) systems, electronic payment machine, and online appointment system, are becoming widely and effectively adopted in reducing the medical treatment seeking time and efforts.

According to above, a successful innovation of medical service depends on accurate decoding the demands from patients, and thereby, the traditional satisfaction assessment about the gaps of treatment benefits and cost is inappropriate [27]. PPV presented a comparative judgment from patients' underlined value: treatment effectiveness, medical service, patient-doctor relationships, and hospital environment, in addition to the expenditures during the treatment seeking process [28, 29]. The augmented medical disputes and patient dissatisfaction in China should secure patients' value perceived in medical treatment seeking, by comparing to paid time and financial costs.

## 3. Methods

Based on the ranking of the Zhejiang Province Health Committee, a twelve-month PPV study on inpatient and outpatient experiences was conducted at 7 well-known hospitals located at four main cities of the Zhejiang Province in China during 2018-2019. A pilot study of 50 interviews was taken to solicit information, from the database of medical dispute claimers from 7 well-known hospitals in Zhejiang Province. The feedback provided initial information and give suggestions on the attributes' selection in the questionnaire. Fifty-seven items from seven dimensions of Perceived Value Theory were consisted in the questionnaires to evaluate patients' satisfaction with medical treatment. Basic information about patients' characteristics would be collected, such as illness states and treatment risks (self-assessment), prepared time in hospitals, the costs of time and expenses, revisit rate, and sought acquaintance before seeking hospital or doctors. Then, patients' historical negative experiences would be requested, such as convenient and comfort environment in treatment, normalization and standardization of medical treatment, communication process and time with doctors, doctor-patients' relationships, reputation, and goodwill of doctors and hospitals.

Subsequently, survey questionnaires were modified and distributed via on-site face-by-face approaches to explore the comprehension of PPV. Demographic information of patients was firstly put in the questionnaire; perception assessment items were placed to invite respondents (patients) to weight their selection (five Likert scale: 1 meant the least important and 5 meant the most important) and open questions regarding other necessary values in assessment. Patients were required to differentiate their selection according to their individual medical treatment seeking experiences. The SPSS statistic software was adopted in data analysis. Seven constructs that consisted of 35 identified items became the finalized 7 constructs, which covered the medical normalization, price, communication, comfort, convenience, hospital reputation, and treatment effectiveness, as shown in Table 1. Then, 3500 questionnaires were equally sent to the 7 hospitals. Patients from outpatient and inpatient departments were given the questionnaires face-by-face. 2586 questionnaires were returned. 53% of the questionnaires were from inpatient regions, and 47% were gathered from outpatients. Valid feedback presented male patients (43%) and female patients' viewpoints (57%).

## 4. Results

Overall satisfaction assessment was presented in Table 1. It indicated a great proportion of patients “dissatisfaction was from hospitals” functional values, covering medical diagnosis and treatment's effectiveness, treatment processes' transparency and standardization, accessibility and convenience, accurate prices, and reasonable charging. Emotional values also played an important role in patients' perception, including sound communication and attitudes from doctors/nurses, comfortable environment, and well facilitates. Furthermore, hospital reputation and medical skills were significant as well in medical treatment seeking, was regarded as social values.

After considering patients' background characteristics of ages, gender, household income, and education level, it displayed a significant deviation for the variables in patients' functional value and emotional value, as exhibited in Table 2. From the demographic analysis of responders' overall valuation scores, younger patients provided lower feedback than aged (*F* = 13.757, *P* < 0.01), male patients held more favorable attitude than females (*F* = 5.523, *P* < 0.01), and inpatients showed better perception than patients from outpatients (*F* = 147.8, *P* < 0.01). Moreover, significant differences also remained in responders' occupation (*F* = 2.367, *P* < 0.05), income level (*F* = 2.597, *P* < 0.05), and education level (*F* = 7.314, *P* < 0.05). The comments from these patients with “business and service” field reflected showed the most negative measurement, while the occupation of “officers” offered the best valuation. The lowest scores came from the group of households' incomes between 3001 and 5000 RMB (monthly), but the rest income groups did not show a considerable difference in overall appraisal. Patients' residency, no matter from the places of rural, town, or urban, did not significantly affect the results of satisfaction appraisal, neither related to medical service convenience and waiting time.

Furthermore, the descriptive statistics displayed (Table 3) patients' differentiated concerns of treatment effectiveness, waiting time, and convenience by comparing to their overall satisfaction evaluation. There were significantly different impacts of the education levels, ages, genders, and patients' sources (inpatients/outpatients) on the patients' perceived value of “treatment effectiveness,” respectively, taking *F* = 3.168, 12.195, 3.388, 197.7, *P* < 0.05. For more details, the group of higher educated male patients in the “60 age and above” in inpatients presented an upper appreciation on the treatment effectiveness than others. In contrast, the group of patients from 19 to 29 age contains the lowest emphasis on treatment effectiveness. About the “convenience” perceived in medical seeking, the bracket of age (*F* = 10.677, *P* < 0.01), gender (*F* = 5.374, *P* < 0.01), income (*F* = 2.639, *P* < 0.05), occupation (*F* = 2.418, *P* < 0.01), education levels (*F* = 10.472, *P* < 0.01), and patients' source (inpatients and outpatients, *F* = 96.18, *P* < 0.01) donated significant difference. Additionally, these attributes in the perceptions “convenience” and “waiting time” in medical treatment seeking illustrated a reasonable degree impacted by patients' characteristics (*F* = 0.371, *P* < 0.01; *F* = 0.487, *P* < 0.01). The overall assessment of satisfaction has a positive relationship with “waiting time” (*F* = 0.397, *P* < 0.01) but not relevant to the convenience significantly (*P* = 0.482). The statistic outcomes recovered that there was no significance in the “waiting time” between females and males but significant in different patients' sources (inpatients and outpatients, *F* = 87.25, *P* < 0.01), ages (*F* = 13.914, *P* < 0.01), education levels (*F* = 22.474, *P* < 0.01), residence place (*F* = 3.18, *P* < 0.05), monthly income levels (*F* = 7.7.472, *P* < 0.01), and occupations (*F* = 2.675, *P* < 0.01). Furthermore, by grouping the respondents in the item of time adequacy, neither the perception of treatment effectiveness (*P* = 0.943 > 0.05) nor the assessed overall satisfaction (*P* = 0.203 > 0.05) had significant correlation to the adequate time for doctors in medical treatment seeking.

## 5. Discussion

The survey carried out a profound thinking about why dissatisfaction is an ordinary occurrence in Chinese hospitals. It created this research's primary interest about the diverse influences on patients' satisfaction levels and their perceived values in medical treatment seeking. As reflected by tradition studies, the main factor influencing satisfaction rate concerns the medical expenses and functional levels of treatment [15] regardless of patients' income level, occupation, or other demographic difference. The speedy growth of the economy development and advanced living standards upgraded Chinese people's expectations of healthcare quality. With the increase in living standards comes the increase in the expectations and perceived value of medical care. At the other side, high-level medical recourses are inadequate to fulfil the vast quantity of population. This medical demanding and affording discrepancy situations resulted distinct patients' satisfaction and perceived values in China.

Learned from the characteristics of Chinese patients in this research, PPV would be affected by the patients' backgrounds, finally influence the evaluation of medical values and patients' satisfaction from various dimensions. Male patients showed more consideration than females in the values of medical treatment, prices, and convenience. Female and young patients scored superior of emotional value and were sensitive to the doctors/nurses' attitudes and comfortable environment. Those highly educated patients put more weight on social value (hospital reputation) but usually hold relatively low satisfaction in emotional values. One explanation came from the higher education levels of patients in big cities with higher social levels and higher income levels but may have lesser time in medical treatment seeking.

It is another interesting result revealed that the sufficiency of treatment time with doctors was not highly emphasized by patients. In other words, even though doctors provided adequate time with patients, their mood remained negative after a long wait. It possibly because patients considered these recognized hospitals and doctors had sophisticated professional and advanced equipment. Therefore, for general medical treatment issues, patients less considered the adequacy of treatment time when they have high trust levels of the quality and reputation of hospitals and doctors. Additionally, a conventional consensus of the heavy workloads and crowed queues in outpatients, particularly in big hospitals, making patients tolerable to the limited communication and time with doctors.

Additional finding of this research was the importance of reasonable waiting time in patients' perceived value. Specially, these patients whose occupations deemed to be busy with high income level (such as technicians and business people) have higher dissatisfaction rate. Urban patients are more sensitive than suburban patients in waiting, when they need consider the traffic or other expenditure due to the time delay. Patients, in the age of 60 and older, have time and thus put light weight about the waiting time. Conversely, younger patients contained low satisfaction due to their tight work schedule, particularly in the age of “18-29” and “30-39” groups. Patients with higher education and income are more likely to be dissatisfied compared with others. Education also determines the patient's way of thinking and value judgment and causes satisfaction differences. Higher education levels usually have more knowledge and capabilities to link the waiting time to inefficiency and unreasonable design of the hospital operation. Outpatients scored lower on waiting time than inpatients, and the reason maybe the inpatients have sufficient time expectation in the hospital. This finding showed an advantage to organize patients' time perception and pass the reasonability of waiting time, as well as reduce the total time spending in treatment waiting.

Convenience is the supplementary perspective of dissatisfaction. In medical treatment seeking, people living in different districts did not illustrate significant differences in estimating the value of convenience; nevertheless, there were still significant discrepancies in inpatients and outpatients, gender, age, education levels, income, and occupation difference. The result also found that male and elder patients (above the ages of 50) highly remark the importance of convenience. Outpatients were likely to present negative reactions to the weak accessibility and convenience than inpatients. An explanation would come from that there were more treatment processes and transfers in outpatients, including stops for registration and decentralized appointments and test location, medicine payment and receiving, and prescription and test report preparing. Particularly for the first in a hospital, unclearness and unfamiliarity of the guiding caused more anxieties and troubles in outpatients. The patient-friend environment and medical treatment seeking processes in outpatient should be redesigned to further enhance the convenience of medical service and reasonability of layout, such as EMR (Electronic Medical Record), automatic payment system, eligible guide service, explicit signs, and relaxed waiting room environment.

Communication was perceived as a significant value in this study, no matter in outpatients or inpatients. The problem was that doctors and hospitals were less sensitive to patients' emotional experiences greatly because they primarily concentrated on medical techniques and device improvement rather than communication skills and relationship management capabilities. Doctors and nurses' attitudes kindly could influence the emotion during or after the treatment. Doctors and nurses usually have more time and opportunities to understand inpatient conditions, and consequently, the communication and relationships placed in a higher satisfaction level than in outpatients. Furthermore, different conditions of illness influenced the satisfaction evaluation: patients who are in heavy health conditions respond more negatively than light illnesses; patients with mild health conditions are usually in a better mood in communication. The patients perceived value of communication did affect the emotional value but has little influence on the functional value of treatments' effectiveness.

A deeper understanding of the patients and their medical values' expectations will accurately improve hospital medical satisfaction via providing patients' suitable personalized service or facilitating according to their distinct groups, such as inpatients and outpatients, different ages, place of residency, education levels, and occupations. Satisfaction of medical service and experiences of interaction in hospitals can be certainly improved based on the highly highlighted perceived value of patients. It could be advantageous medical care improvement projects to construct classified satisfaction management modes, basing on a well understanding of differentiated weights from the characteristics of patients and differentiated perceived value. In this case, a sound perceived value concentrated system is about matching the degree of hospital convenience and communication environment with patients' background characteristics. These characteristics influenced the preferences in patient-perceived values and reach a differentiated patients' satisfaction. Hospitals should adopt a substantial database and supportive information mechanisms to gather patients' information and then redesign categorized medical treatment seeking processes. For example, those patients who are well educated or young with the e-technologies adaption abilities, can be encouraged to experience self-assistant intelligent facilities or AI prediagnosis. These online medical systems incredibly assist the convenience, waiting time control, communication in treatment service.

## 6. Conclusion

Patients' dissatisfaction and medical disputes reflected a gap between the hospitals' perception and patients' expectation in China. This research targeted on how to manage satisfaction from patient-perceived values. PPV analysis discussed the importance of enhancing medical care service satisfaction via psychological management. According to the 2586 questionnaires collected from 7 well-known hospitals located at four main cities of the Zhejiang Province in China in 2018-2019, the results of analysis provide further initiatives to examine patients' characteristics and dissimilar impacts on their perceived values as well as the degrees of satisfaction levels in medical treatment seeking. This research deepens the understanding that patients' satisfaction and dissatisfaction can be significantly reflected by their perceived values, not simply from functional values but also from emotional values and social values. This research added a new perspective by collecting empirical data utilizing control critical confounding factors to distinguishing patients' characteristics on their perceived value, including primary indicators, aspects, actual perceived value, and degree of importance.

Diagnosis and treatment effectiveness unquestionably are the main focus as the perspective of functional value. Inconvenience, uncomfortable crowding, redundant waiting time, and slight communication in medical treatment seeking produced considerable patient dissatisfaction. The valuable analysis placed that Chinese patients' dissatisfaction was significantly affected by their background characteristics, covering the age, gender, income levels, educational levels, and health conditions.

Hospitals in China can adopt categorized patient satisfaction management strategies to improve patients' perceptions of medical value in medical treatment seeking. Considering the circumstances of getting medical treatments, the patients' time pressure and convenient accessibility of service and layout demand a higher efficacy design in hospital without time wasting, especially for these younger (especially for the ages of 19-39), high income, and educated groups. However, the indictor description and questionnaire design instruction not fully explained which may cause the patients not fully understanding the questions and affect the reliability of the results. Especially under the COVID-19 circumstance, any changes or difference in PPV would be valuable for further study.

## Figures and Tables

**Table 1:** Demographic analysis of patients' perceived value.

Aspects	Indicators		Numerical value			
	Primary indicators	Secondary indicators	Actual perceived value	Degree of importance	Importance of primary indicators	Importance of aspects
Functional value	Treatment effects	Effect	3.76	4.16	4.14	3.91
		Diagnosis	3.98	4.54		
	Prices	Reasonability of prices	3.52	4.06	3.96	
		Accuracy of bills	3.89	4.07		
	Normalization	Standardization	3.95	4.18	3.92	
		Transparency	4.00	3.83		
	Convenience and accessibility	Reasonability of layout	3.65	3.82	3.61	
		Convenience of medical service	3.79	3.75		

Emotional value	Communication	Doctors' attitude	4.03	4.21	3.97	3.92
		Nurses' attitude	4.06	4.05		
	Comfort	Environmental hygiene	3.78	3.94	3.87	
		Completion of supporting facilities	3.84	3.93		

Social value	Hospital reputation	Advanced medical equipment	4.18	3.84	3.86	3.86
		Influence of medical skills	4.40	4.13		

(1) The secondary indictors only showed the most important two; (2) “Importance of aspects” was average values of “Importance of Primary indicators,” and “Importance of Primary indicators” was average values of “Importance of secondary indicators.”

**Table 2:** Differentiated perceived values from patients' varied characteristics.

Patient background features	Differentiation of characteristics		Relationships with characteristics		Degree of perceived value (high or low) and patients' features	
	Emotional value	Functional value	Emotional value	Functional value	Emotional value	Functional value
Outpatients/inpatients	Sig	Sig	+	+	High for inpatients Low for outpatients	High for inpatients Low for outpatients
Illness condition	Sig	Sig	-	-	Negative relationship with illness condition	Negative relationship with illness condition
Gender	Sig	Sig	+	-	High for men Low for women	High for men Low for women
Age	Sig	Sig	+	+	Positive relationship with age	Positive relationship with age
Educational level	Sig	Sig	-	-	Negative relationship with education degree	Negative relationship with education degree
Monthly income	Sig	None	-	None	Negative relationship with income	None

The relationship is as follows: +: relatively high; -: relatively low; ++: significantly high; --: significantly low; 0: no difference (*P* > 0.05).

**Table 3:** Patients' differentiated satisfaction levels in cooperation with perceptions of waiting time, convenience, and treatment effectiveness.

Feature	Groups	Proportion of patients	Overall assessment		Perception of waiting time		Perception of convenience		Perception of treatment effect	
			$\bar{x}\pm s$	*F*	$\bar{x}\pm s$	*F*	$\bar{x}\pm s$	*F*	$\bar{x}\pm s$	*F*
Patients' source	Inpatients	53%	4.08 ± 0.70	147.8^∗∗^	3.55 ± 0.96	87.25^∗∗^	3.79 ± 0.82	96.18^∗∗^	3.99 ± 0.78	197.7^∗∗^
	Outpatients	47%	3.76 ± 0.70		3.20 ± 1.0		3.48 ± 0.83		3.56 ± 0.79	

Gender	Male	43%	3.99 ± 0.71	5.523^∗∗^	3.40 ± 1.0	0.36	3.72 ± 0.82	5.374^∗∗^	3.84 ± 0.82	3.388^∗^
	Female	57%	3.89 ± 0.72		3.37 ± 0.99		3.59 ± 0.84		3.75 ± 0.80	

Age	19-29	33%	3.80 ± 0.69	13.757^∗∗^	3.20 ± 1.03	13.914^∗∗^	3.63 ± 0.81	10.677^∗∗^	3.63 ± 0.80	12.195^∗∗^
	30-39	22%	3.89 ± 0.73		3.29 ± 1.01		3.79 ± 0.79		3.79 ± 0.79	
	40-49	14%	4.01 ± 0.70		3.52 ± 0.92		3.87 ± 0.80		3.87 ± 0.80	
	50-59	10%	4.10 ± 0.66		3.58 ± 0.90		3.97 ± 0.77		3.97 ± 0.77	
	60 and older	13%	4.13 ± 0.68		3.65 ± 0.93		3.98 ± 0.80		3.98 ± 0.80	

Residence place	Urban area	35%	3.93 ± 0.72	0.081	3.32 ± 0.97	3.18^∗^	3.63 ± 0.81	0.472	3.81 ± 0.81	0.869
	Town	26%	3.94 ± 0.70		3.43 ± 0.98		3.65 ± 0.84		3.75 ± 0.81	
	Rural area	39%	3.92 ± 0.72		3.41 ± 1.02		3.66 ± 0.86		3.79 ± 0.80	

Education level	Primary school	16%	4.00 ± 0.70	7.314^∗^	3.56 ± 1.02	22.474^∗∗^	3.77 ± 0.8	10.472^∗∗^	3.86 ± 0.81	3.168^∗∗^
	High school	34%	4.00 ± 0.72		3.54 ± 0.96		3.73 ± 0.84		3.83 ± 0.83	
	College school	25%	3.85 ± 0.72		3.31 ± 0.95		3.58 ± 0.81		3.74 ± 0.80	
	Undergraduate	24%	3.85 ± 0.69		3.12 ± 1.02		3.52 ± 0.83		3.72 ± 0.77	

Income per month (RMB)	500-1500	22%	3.98 ± 0.68	2.597^∗^	3.49 ± 0.98	7.472^∗∗^	3.72 ± 0.87	2.639^∗^	3.78 ± 0.83	1.395
	1501-3000	34%	3.93 ± 0.70		3.37 ± 0.95		3.63 ± 0.80		3.76 ± 0.78	
	3001-5000	22%	3.86 ± 0.71		3.32 ± 1.02		3.61 ± 0.84		3.76 ± 0.79	
	5001 and above	22%	3.94 ± 0.76		3.22 ± 1.03		3.59 ± 0.86		3.86 ± 0.84	

Occupation	Officer	12%	3.90 ± 0.70	2.367^∗^	3.36 ± 0.97	2.675^∗∗^	3.64 ± 0.77	2.418^∗∗^	3.78 ± 0.80	1.564
	Self-employed	14%	3.94 ± 0.66		3.37 ± 0.98		3.62 ± 0.86		3.78 ± 0.80	
	Student	10%	3.89 ± 0.73		3.27 ± 1.11		3.61 ± 0.89		3.75 ± 0.82	
	Technician	8%	3.93 ± 0.71		3.22 ± 0.9		3.54 ± 0.84		3.72 ± 0.83	
	Farmer	17%	3.98 ± 0.71		3.53 ± 1.02		3.79 ± 0.88		3.85 ± 0.82	

(1) The secondary indicators only showed the majority of investigated patients; (2) ^∗^*P* < 0.05, ^∗∗^*P* < 0.01.

## Data Availability

The data about the findings of this study are available from the corresponding author upon reasonable request.

## Abbreviations

PPV: Patient Perceived Value
EMR: Electronic Medical Record.
